# Do Novice Runners Show Greater Changes in Biomechanical Parameters?

**DOI:** 10.1155/2021/8894636

**Published:** 2021-01-04

**Authors:** Wenjing Quan, Feng Ren, Dong Sun, Gusztáv Fekete, Yuhuan He

**Affiliations:** ^1^Faculty of Sports Science, Ningbo University, China; ^2^Savaria Institute of Technology, Eötvös Loránd University, Hungary

## Abstract

**Purpose:**

Examining and understanding the biomechanics of novice runners and experienced runners can further improve our knowledge within the field of running mechanics and running injuries. The purpose of this study was to classify the differences in lower limb biomechanics during a 3.3 m/s running task among both experienced runners and novice runners.

**Method:**

Twenty-four participants (12 experienced runners and 12 novice runners) ran at 3.3 m/s across a force plate; kinematics and kinetics data were collected by the Vicon motion system and Kistler force plate. Group comparisons were made using an independent samples *t*-test to identify differences in the impact peak, loading rate, contact time, ankle, knee, and hip joint kinematics and kinetics during the stance phase.

**Results:**

No significant differences were observed between novice and experienced runners for both ankle and knee joint kinetics except that the ankle joint plantar flexion torque was significantly greater in the novice runners. However, the plantar flexion, dorsiflexion, range of motion (ROM), plantar flexion torque, and max angular velocity of ankle joint significantly increased in novice runners than inexperienced runners. Additionally, the flexion angle and range of motion of the hip joint were observed to be larger in the novice runners. Moreover, the maximum extension torque and the maximum extension power in the hip joint were significantly increased in the experienced runners. There were no significant differences in the first peak, contact time, and average vertical loading rate. Novice runners showed a larger vertical instantaneous loading rate than experienced runners.

**Conclusion:**

These preliminary findings indicate that novice runners are prone to running injuries in comparison to experienced runners. Novice runners showed larger kinematics and kinetic parameters in the joint of the ankle and hip. Novice runners should enhance muscle strength in the hip and choose scientific training methods.

## 1. Introduction

Running is one of the most popular recreational physical activities in the world. Regular running helps prevent the incidence of chronic diseases, such as cardiovascular disease and obesity [1, 2]. Because of easy accessibility, many people prefer participating in long-distance running which can increase cardiopulmonary function and relieve psychological stress [3]. Unfortunately, excessive running can trigger running-related injuries and musculoskeletal injuries to develop [4, 5]. Running injuries are mainly lower limb injuries, primarily knee joint injuries, especially in the front of the knee (such as patellofemoral joint pain) [6–8]. Other common injuries include strains of the tibia, Achilles tendon, gastrocnemius, foot, and thigh muscles [4].

A previous study has shown that the risks of overuse running injury were increased from 20% to 70% in recreational and competitive distance runners [9]. Videbæk et al. have demonstrated the incidence of injury per 1000 hours of running, in which the rate of injury was 17.8% of novice runners compared to recreational runners (7.7%) and ultramarathon runners (7.2%) [10]. Of all populations, novice runners experience a high rate of injury. Novice runner's injury rate was higher compared to recreational, competitive, or marathon runners [11]. It is important to focus on injury prevention among novice runners. Nevertheless, there are few research recommendations for novice runners who desire to begin running training. There are many reasons which can cause running injuries, such as error training, the difference in running surface, different running habits, and running shoes [12, 13]. Although scientific researchers and clinical staff have been working hard to help runners reduce running-related injuries, the incidence of injuries has remained high for many years [14].

Epidemiological studies have found that overuse injuries were associated with kinematic variables of lower limb joints: the increased hip interrotation and hip adduction [13, 15]. Novacheck also found that the increased eversion angle velocity and ankle eversion angle might trigger the development of overuse injuries (Sallis et al., 1992). Running-related injuries were associated with ground reaction force, specifically increased vertical loading rate and vertical instantaneous loading rate, and the first peak caused the tibial stress fractures [16].

Running-related injuries especially in the knee joint have the characteristics of the frequent occurrence in people without running experience [17, 18]. Psychological fear of running-related injuries makes it difficult for nonrunning habit groups to form running habits [19], which hinders the widespread development of running.

Thus, several studies show a biomechanical difference between novice and experienced runners. Schmitz et al. found that there were no significant differences in impact peak, loading rate, peak nonsagittal hip kinematics, or strength among the novice runners and competitive runners. However, novice runners showed larger peak hip internal rotation and a decrease in trunk side-plank endurance [20]. When novice runners and competitive runners ran in a state of fatigue, novice runners showed larger hip abduction and peak trunk lean during midswing [21]. Van Mechelen proposed that about 50% to 75% of sports injuries may be due to overuse injuries caused by the repeated repetition of the same action. Factors related to running injuries include a history of previous sports injuries, a lack of running experience, participation in running competitions, and running long distances per week [22]. Moreover, the effect of running experience on the kinematics and kinetic energy of the lower limb remains unclear. Thus, the purpose of this study was to determine the effect of running experienced on lower limb biomechanical changes during the stance phase at 3.3 m/s among both experienced runners and novice runners. The hypotheses were that the novice runners' group would show higher changes in kinematics and kinetics when compared with experienced runners.

## 2. Methods

### 2.1. Participants

Two populations were recruited using flyers around the society and university: experienced runners and novice runners. The experienced runners consisted of 12 males that had been running at least 20 miles per week and the running experience was more than 5 years. The novice runner consisted of 12 males who ran 2 or 5 miles per week. A novice runner was defined as an individual having no former experience in running and never taken part in a running competition. All information about the 24 endurance runners is given in Table 1. Only subjects having the target foot length of US size 9 (±0.5) and self-reported as right leg dominant (defined as the preferred kicking leg) were included. Exclusion criteria consisted of any spinal or lower extremity surgery or any knee ligament or cartilage pathology in the past year. For this test, all the participants were rearfoot strikers (RFS) [23]. Written informed consent was obtained from the subjects, and the testing procedures were approved by Ningbo University.

### 2.2. Biomechanical Modeling and Collecting

An eight-camera motion analysis system (Vicon, Metrics Ltd., Oxford, UK) was used to capture the sagittal plane kinematics of the dominant lower extremity at a frequency of 200 Hz [24]. Participants were required to wear tight-fitting pants and T-shirts. All subjects ran with the right foot stepping on a single embedded force plate (Kistler Type, 9281B, Kistler Instrument AG, Winterthur, Switzerland) with dimensions of 600 × 900 mm, which was fixed in the middle of the 15 m walkway and was utilized to collect the ground reaction force (GRF) at a frequency of 1000 Hz. The heel strike and toe-off were determined when the vertical GRF crossed a 30 N threshold level [21]. Kinematic data were collected including angle changes of the lower limb joints (hip, knee, and ankle) in sagittal planes during the stance phase. Kinetic parameters were ground reaction force, joint moment, and joint power.

Retroreflective markers were placed on the subjects according to previous research which included thigh, shank, and ankle [25] (Figure 1). Twenty-five retroreflective markers (diameter: 14.0 mm) were used to define the knee, ankle, and hip segments. The marker locations included right and left anterior superior iliac spine, left and right posterior superior iliac spine, right and left greater trochanter, first and fifth metatarsal heads, distal interphalangeal joint of the second toe, medial and lateral malleoli, and medial and lateral epicondyle of the femur; tracking clusters were placed on the lateral thigh, shank, and right heel (Table 2).

### 2.3. Running Protocol

All participants wore the same type of running shoe, Anta (Flashedge, China). Participants were instructed to warm up with light jogging and stretching in the common shoes. They then ran for at least 5 minutes in the laboratory at a self-generated comfortable speed. Runners performed each trial by running through a laboratory that was 15 m long and exiting into a hallway. On both sides of the force platform was a speed-measuring instrument (smart speed, Fusion Sport Inc., Burbank, CA, USA) to control the speed of the subjects. The distance between the speed-measuring instrument was 3.3 m. All the subjects ran at a speed of 3.3 m/s. Each test collected six successful trials (Figure 2).

### 2.4. Data Analysis

This study paid more attention to the variation of the sagittal plane as the main data [26]. Visual 3D (C-motion, Germantown, MD, USA) was used to process the data. First, a fourth-order low-pass zero-lag Butterworth filter was used to filter the marker trajectories at 15 Hz and force plate data at 100 Hz [26].

Sagittal plane hip, knee, and ankle angles were calculated using Cardan angles with the distal segment expressed relative to the proximal segment in Visual 3D. The net internal joint moments and joint powers were calculated using a standard inverse dynamics approach. Segment masses, the center of mass locations, and inertial properties were calculated for the thigh, shank, and foot using anthropometric data [27]. The joint kinetic and the GRF variables were normalized by the subject's body mass. Joint angles, joint moments, and powers were normalized to the stance phase over 101 data points. Max angles were defined as the maximum joint angle during the stance phase, while participants ran the 15 m distance. Min angles were defined as the minimum joint angle during the stance phase. The range of motion was defined as the maximum angle minus the minimum angle. The average vertical loading rate (VALR) and vertical instantaneous loading rate (VILR) were calculated over the portion of the vertical GRF (vGRF) vs. time curve between 20 and 80% of the time to peak impact according to Equations (1) and (2) (Milner et al., 2008).

(1) $$\begin{array}{c} \text{VALR}=\frac{F_{80}\%-F_{20}\%}{t_{80}\%-t_{20}\%}, \end{array}$$

(2) $$\begin{array}{c} \text{VILR}=\frac{\Delta F_{\max}}{\Delta t}\text{ where }\left(t_{20}\%<t<t_{80}\right), \end{array}$$

Kinematic variables of two groups of runners included eversion and dorsiflexion angles (ankle, knee, and hip), as well as joint (ankle, knee, and hip) angle velocity in the sagittal plane (Figure 3). Kinetic variables included contact time, average vertical loading rate (VALR), vertical instantaneous loading rate (VILR), first peak, joint moment, and joint power.

### 2.5. Statistical Analysis

All data are given as mean ± standard deviation. Normal distribution and homogeneity were assessed using the Shapiro-Wilk test and Levene's test, respectively. Using SPSS (SPSS Inc., Chicago, IL), an independent samples *t*-test was used to assess group differences for kinematic and kinetic parameters. The level of significance was set to *p* = 0.05.

## 3. Results

### 3.1. Kinematics of Ankle, Knee, and Hip Joints

The Shapiro-Wilk tests revealed that all parameters were normally distributed. There was no significant difference in the max knee angular velocity, min hip angle, and max hip angular velocity. When analyzing the changes in the joint angles of novice runners during the stance phase (Table 3), maximum ankle angle (*p* < 0.01), minimum ankle angle (*p* < 0.05), ROM of ankle joint (*p* < 0.01), maximum hip angle (*p* < 0.01), ROM of the hip joint (*p* < 0.01), and ROM of knee joint (*p* < 0.01) were increased. In addition, decreased changes were observed in the maximum knee angle (*p* < 0.01) and minimum knee angles (*p* < 0.01) in the novice runners (Figure 4).

### 3.2. Kinetics of Ankle, Knee, and Hip Joints

Minimum moment of the hip joint (*p* < 0.05) and the maximum power of the hip joint (*p* < 0.05) were significantly smaller in the novice runners than in the experienced runners (Table 4). The minimum ankle moment was significantly greater in the novice runners than in the experienced runners (Table 4) and (Figure 5). However, there were no significant differences in the maximum moment, maximum power, minimum power of ankle joint, maximum moment, and minimum power of hip joint. No significant differences existed in the kinematic parameters of the knee joint (Table 4).

### 3.3. Kinetics of Ground Reaction Force

Contact time increased significantly among novice runners compared to the experienced runners (*p* < 0.01) (Table 5). No significant difference was observed in the vertical average loading rate, contact time, and first peak. Besides, the vertical instantaneous loading rate was lower in the novice runners in comparison to the inexperienced runners (*p* < 0.01).

## 4. Discussion

Future research directions may also be highlighted [28, 29]. Compared with the ankle variables, the plantar flexion, dorsiflexion, ROM, plantar flexion torque, and maximum angular velocity were significantly increased in novice runners when compared to inexperienced runners. Long-distance running may cause plantar fasciitis and metatarsal stress fracture-related running injuries.

A previous epidemiological investigation found that the knee joint of novice runners is the most prone to injury [30]. Our study results showed that the maximum knee angle and minimum knee angles were smaller than experienced runners. Dierks et al. found that increased knee flexion helps reduce the risk of a knee injury. However, in this study, novice runners observed larger knee flexion than experienced runners [31]. The ROM of the knee joint was larger in the novice runners than experienced runners, and this finding is in agreement with Agresta et al. [32]. This could be attributed to novice runners having poor running mechanics, which results in higher loads on musculoskeletal tissue, especially at the tibia and the knee.

The novice did show greater hip joint flexion angle and ROM of the hip joint in this study. The hip joint plays a very important role in the movement of the lower limbs, and the instability of the hip joint is considered to be an important mechanism of lower limb injuries [9]. In the sagittal plane, the novice runners produced a larger ROM in comparison to the experienced runners. This may suggest poor hip stability among novice runners. The maximum extension torque and the maximum extension power in the hip joint significantly increased in the experienced runners. This phenomenon might have been caused by running miles and running speed. In addition, insufficient hip abductor muscle strength and abnormal anatomical force lines may also affect it [9, 33]. Also, larger extension torque and extension power in the hip joint might lead to the development of iliotibial bundle friction syndrome.

The curve of the ground reaction force during running is a typical double-peak curve. Studies suggest that the increase in the ground reaction force peak and its loading rate will cause higher risks to lower limb injuries [34–36]. In this study, the peak ground reaction force and the corresponding average load rate of the ground reaction forces were consistent with the results of Schmitz et al., who used the same test speed in their experiments [20]. However, the vertical instantaneous loading rate was lower in the novice runners. Many factors may influence the ground reaction force parameters.

Although the ground reaction force parameters were associated with running injuries, our results do not provide more details into novice runners who have a higher rate of running injuries than experienced runners. For novice runners, the risk of running injury was higher than experienced runners. Novice runners should enhance muscle strength in the hip and choose scientific training methods. During the training sessions, novice runners should increase the amount of running and control the running speed on a step-by-step basis and reasonably.

There are some potential limitations to this study. In this study, the anteroposterior ground reaction force was not calculated. The data of anteroposterior ground reaction force might provide a helpful understanding of overuse running injuries for both novice and experienced runners. Moreover, the different running speeds should be considered when compared to the biomechanics parameters. Finally, a further study should focus on the effect of different gender and different BMI.

## Figures and Tables

**Figure 1:** Placement of combined marker set consisting of retroreflective cluster markers and single 14 mm retroreflective markers.

**Figure 2:** Participant motion capture setup.

**Figure 3:** Pictorial illustration of the running gait cycle during the stance phase at 3.3 m/s.

**Figure 4:** Sagittal ankle, knee, and hip joint kinematics for novice runners (the solid blue line is the mean and the shaded area is the standard deviation) and experienced runners (dashed red line is the mean). Note: the dotted box indicates a significant difference between the two groups of runners, *p* < 0.05.

**Figure 5:** Sagittal ankle, knee, and hip joint power and moment for novice runners (the solid blue line is the mean and the shaded area is the standard deviation) and experienced runners (dashed red line is mean). Note: the dotted box indicates a significant difference between the two groups of runners, *p* < 0.05.

**Table 1:** The basic demographics of subjects (*n* = 24).

Characteristic	Experienced	Novice
Age (years)	26.20 ± 4.10	25.60 ± 4.70
Weight (kg)	63.40 ± 7.50	67.50 ± 6.80
Height (cm)	170.00 ± 8.28	173.00 ± 7.28
BMI (kg/m^2^)	21.75 ± 2.60	22.89 ± 3.20
Running experience (years)	5.20 ± 3.00	2.10 ± 1.60

**Table 2:** Anthropometric data.

Segment	Definition	Center of mass (%)	Radius gyration (%)
Foot	Lateral malleolus/head metatarsal II	1.37	4.415
Shank	Femoral condyles/medial malleolus	4.33	4.395
Thigh	Greater trochanter/femoral condyles	14.16	40.95

**Table 3:** Ankle, knee, and hip joint kinematics during the stance phase (*n* = 24).

Joint	Variables	Experienced	Novice	*p* value
Ankle	Max angle (°)	8.20 ± 1.60	23.70 ± 1.11	*p* < 0.01∗
	Min angle (°)	−14.51 ± 2.66	−8.20 ± 3.47	*p* < 0.01∗
	ROM (°)	22.72 ± 2.53	31.90 ± 3.89	*p* < 0.01∗
	Max angular velocity (°/s)	180.98 ± 29.20	205.19 ± 15.19	0.026^∗^

Knee	Max angle (°)	−7.70 ± 3.00	−20.50 ± 2.56	*p* < 0.01∗
	Min angle (°)	−32.82 ± 3.01	−49.06 ± 2.09	*p* < 0.01∗
	ROM (°)	25.11 ± 2.98	28.56 ± 4.31	0.041^∗^
	Max angular velocity (°/s)	181.71 ± 33.05	205.86 ± 63.13	0.277

Hip	Max angle (°)	26.07 ± 2.89	32.69 ± 2.15	*p* < 0.01∗
	Min angle (°)	−1.63 ± 4.98	−2.58 ± 2.90	0.059
	ROM (°)	27.71 ± 4.10	35.27 ± 2.57	*p* < 0.01∗
	Max angular velocity (°/s)	19.11 ± 18.64	21.91 ± 45.06	0.851

Note: ^∗^significant difference between experienced runners and novice runners (*p* < 0.05).

**Table 4:** Ankle, knee, and hip joint kinetics during the stance phase (*n* = 24).

Joint	Variables	Experienced	Novice	*p* value
Ankle	Max moment (Nm)	0.50 ± 0.24	0.43 ± 0.14	0.356
	Min moment (Nm)	−1.85 ± 0.32	−2.22 ± 0.11	0.002^∗^
	Max power (W/kg)	10.43 ± 2.87	11.44 ± 2.35	0.379
	Min power (W/kg)	−3.15 ± 0.85	−4.03 ± 0.77	0.018

Knee	Max moment (Nm)	0.93 ± 0.23	1.08 ± 0.44	0.379
	Min moment (Nm)	−2.71 ± 0.22	−2.63 ± 0.27	0.295
	Max power (W/kg)	1.02 ± 0.43	1.15 ± 0.58	0.530
	Min power (W/kg)	−9.52 ± 2.36	−9.16 ± 1.87	0.681

Hip	Max moment (Nm)	0.82 ± 0.24	0.80 ± 0.12	0.747
	Min moment (Nm)	−4.37 ± 0.45	−3.67 ± 0.48	0.002^∗^
	Max power (W/kg)	17.09 ± 2.81	12.45 ± 3.30	0.002^∗^
	Min power (W/kg)	−1.24 ± 0.60	−1.15 ± 3.26	0.748

Note: ^∗^significant difference between experienced runners and novice runners (*p* < 0.05).

**Table 5:** Ground reaction force parameter during the stance phase (*n* = 24).

Parameter	Experienced	Novice	*p* value
Contact time (ms)	231.00 ± 11.97	230.00 ± 11.97	0.67
Vertical average loading rate (BW/S)	52.58 ± 15.78	48.13 ± 3.60	0.405
Vertical instantaneous loading rate (BW/S)	106.13 ± 41.53	89.00 ± 9.96	0.001^∗^
First peak (BW)	2.15 ± 0.20	2.45 ± 0.18	0.852

Note: ^∗^significant difference between experienced runners and novice runners (*p* < 0.05).

## Data Availability

The data that support the findings of this study are available from the corresponding author upon reasonable request.
